This article has been retracted.

# The Value of DTI Parameters in Predicting Postoperative Spinal Cord Function Fluctuations in Patients with High Cervical Disc Tumors

**DOI:** 10.1155/2022/4957275

**Published:** 2022-03-19

**Authors:** Lin Wang

**Affiliations:** Department of Neurosurgery, The First Affiliated Hospital of USTC, Division of Life Sciences and Medicine, University of Science and Technology of China, Hefei, Anhui 230036, China

## Abstract

**Objective:**

To explore the characteristics of magnetic resonance diffusion tensor imaging (DTI) parameters in patients with high cervical spinal myeloma and the evaluation of postoperative spinal cord function.

**Methods:**

In recent years, 42 patients with high cervical spine myeloma were selected as the observation group, and 42 healthy volunteers were selected as the control group during the same period. The apparent dispersion coefficient (ADC), the fractional anisotropy (FA), the number of fiber bundles (FT), and the fiber bundle ratio (FTR) were compared between the two groups. The correlation between the ADC, FA, FT, FTR, and the International Standard for Neurological Classification of Spinal Cord Injury (ISNCSCI) score in the observation group were analyzed. Spinal cord function was evaluated using the Japanese Orthopaedic Association Score (JOA). Logistic regression model was used to analyze the factors affecting the recovery of spinal cord function after surgery. The receiver operating characteristic curve (ROC) was used to analyze the value of ADC, FA, FT, FTR1, and FTR2 in predicting the recovery of spinal cord function.

**Results:**

The ADCs of the lesion layer and lower layer of the observation group were higher than the middle and lower layers of the control group, the FA and FT were lower than the middle and lower layers of the control group, and FTR1 and FTR2 were lower than those of the control group (*P* < 0.05). The ADC of the lesion layer in the observation group was negatively correlated with ISNCSCI score, and the FA, FT, FTR1, FTR2, and ISNCSCI scores were positively correlated (*P* < 0.05). Three months after the operation, JOA was used to evaluate the spinal cord function, which was excellent in 23 cases and poor in 19 cases. Logistic regression model analysis showed that after the ISNCSCI score was controlled, the increase in ADC and the decrease in FA, FT, FTR1, and FTR2 of the lesion layer were independent risk factors for poor postoperative body function recovery (*P* < 0.05). ROC analysis showed that the combination of ADC, FA, FT, FTR1, and FTR2 of the lesion layer predicted the AUC of spinal cord functional recovery was 0.941, which was better than the single prediction (*P* < 0.05).

**Conclusion:**

The abnormal DTI parameter values of patients with high cervical spinal myeloma can better reflect the lack of spinal cord function, and they can effectively predict the recovery of the patient's body function after surgery, providing a reference for clinical diagnosis and treatment.

## 1. Introduction

Spinal cord tumor refers to tumors occurring in the spinal cord and spinal canal, which can cause spinal cord injury and dysfunction in different degrees. The injury mechanisms include direct destruction of gray matter structure, mechanical compression, and influence on cerebrospinal fluid and blood circulation [1]. The incidence of high cervical spinal cord tumor (C1-C4) is low, but because of its proximity to medulla oblongata, it is difficult to diagnose and treat clinically because of its unique physiological and anatomical characteristics [2]. Surgical resection is the most effective treatment for high cervical spinal cord tumor, but due to the particularity of tumor location, it is easy to leave human dysfunction after operation [3]. Magnetic resonance imaging (MRI) is one of the most valuable noninvasive imaging diagnostic methods for myeloma at present, but conventional MRI cannot show the fine structure of spinal cord, especially the white matter fiber bundle injury, which has certain limitations [4]. Magnetic resonance diffusion tensor imaging (DTI) makes use of the anisotropic characteristics of water molecules in tissues to quantitatively analyze the changes of spinal cord tissue structure and reconstructs the course of white matter fiber bundles by DTI, which provides more valuable information for clinical diagnosis and treatment of myeloma [5, 6]. At present, there is little research on the value of DTI parameters in evaluating the spinal cord function of patients with high cervical spinal cord tumor after operation. Based on this, this study explores the characteristics of DTI parameters of patients with high cervical spinal cord tumor and its value in evaluating postoperative spinal cord function, in order to provide reference for clinical diagnosis and treatment. The report is as follows.

## 2. Materials and Methods

### 2.1. General Information

In recent years, 42 patients with high cervical spinal cord tumor in our hospital were selected as the observation group, and 42 healthy volunteers were selected as the control group in the same period. Inclusion criteria of observation group: patients with high cervical spinal cord tumor were to be diagnosed; no implants or metal foreign bodies in the body; no history of spinal cord or spinal surgery. Inclusion criteria of control group: the control group was matched according to 1 : 1, the principle of matching was that the same spinal cord segment as the observation group was scanned, there was no implant or metal foreign body in the body, there was no central nervous system disease or spinal surgery history, and they were willing to cooperate with the examination. Exclusion criteria: there are serious complications and unstable vital signs; complicated with other central nervous system diseases; cannot cooperate with the inspection. In the observation group, there were 15 males and 27 females, aged from 24 to 75 years, with an average of (46.33 ± 10.51) years, 19 extramedullary tumors and 23 intramedullary tumors; the “spinal cord topographic map” technique was used to identify the posterior median sulcus of the spinal cord, remove the tumors in the spinal cord, and perform laminectomy and laminoplasty according to the condition after operation to prevent spinal deformity. There were 26 males and 16 females in the control group, aged from 24 to 75 years, with an average of (41.25 ± 9.36) years. There is no significant difference in age and sex between the two groups (*P* > 0.05), which is comparable. Patients and healthy volunteers were informed and signed informed consent forms. This study was approved by the hospital's medical ethics committee and was carried out in strict compliance with ethical regulations.

### 2.2. Methods

1. *DTI Parameters*. The general electric company's discovery MR750W 3.0 T magnetic resonance scanner is used. Scanning range: 2 cm above the lesion to 2 cm below the lesion in the observation group, and the same segment of the lesion in the control group and the observation group. Routine sagittal and cross-sectional T2 weighted image scanning, cross-sectional proton density-weighted image scanning, and cross-sectional DTI scanning were performed successively. In the observation group, intravenous injection of paramagnetic contrast agent diethylenetriamine gadolinium pentaacetate (0.1 mmol/kg) was used for T1 weighted image enhancement scanning. The obtained data were imported into AW4.7 software of magnetic resonance workstation for image processing, and the apparent diffusion coefficient (ADC), fractional anisotropy (FA), fiber tract (FT), and fiber tract ratio (FTR) were calculated layer by layer. The ratio of FT of lesion layer to FT of upper and lower lesions in the observation group was FTR1 and FTR2, respectively, and the ratio of FT of middle layer to FT of upper and lower lesions in the control group was FTR1 and FTR2, respectively
2. *Postoperative Evaluation of Spinal Cord Function*. The Japanese Orthopaedic Association Score (JOA) was used to evaluate spinal cord function 3 months after operation, [(postoperative score − preoperative score)/(17 − preoperative score)] × 100% was the functional recovery rate, the functional recovery rate ≤ 50% was poor functional recovery, and the functional recovery rate > 50% was functional recovery

### 2.3. Observation Index

1. Two groups of ADC, FA, FT, and FTR
2. The correlation between ADC, FA, FT, FTR, and international standards for neurological classification of spinal cord injury (ISNCSCI) score in the lesion layer of observation group. ISNCSCI score: sports score: check the muscle function of 10 pairs of sarcomere, and the total score of upper and lower limbs is 50 points; sensory score: check the light touch and acupuncture sensation at the key points of 28 skin joints on the left and right sides of the body, and add the motor score and sensory score as the total score
3. The patient's spine function was evaluated using the JOA scale for 3 months after operation, and the factors affecting spine function were evaluated
4. In order to predict the recovery of spine function, the ADC, FA, FT, FTR1, and FTR2 and JOA scores of the diseased layer were analyzed by ROC regression analysis

### 2.4. Statistical Treatment

The statistical software SPSS22.0 was used to process the data, and the measured data obeyed the normal distribution by Shapiro-Wilk normality test and was described by (*x* ± *s*). Bartlett variance homogeneity test was used to confirm the homogeneity of variance, and independent sample *T* test was used to compare between groups; The data are expressed by *n*(%) and tested by *χ*^2^; Pearson was used to analyze the correlation; Logistic regression analysis was used for influencing factors. The predicted value was analyzed by receiver operating characteristic curve (ROC) curve, and AUC, confidence interval, sensitivity, specificity, and cut-off value were obtained. Logistic binary regression fitting was carried out for joint prediction, and the prediction probability logit (*p*) was returned as an independent test variable. Two-sided test was used, *α* = 0.05.

## 3. Result

### 3.1. Two Groups of ADC, FA, FT, and FTR

The ADC, FA, FT, and FTR of the upper, lower, and lower layers of lesions in the observation group were compared with those in the control group. The results showed that the ADC of the lesion layer in the observation group was higher than that of the middle layer of the control group, while the FA and FT were lower than that of the middle layer of the control group (*P* < 0.05). The ADC, FA, and FT of the lower lesion in observation group were lower than those in control group (*P* < 0.05). The FTR1 and FTR2 in observation group (upper layer of lesion) were lower than those in control group (*P* < 0.05), see Table 1.

### 3.2. The Correlation between ADC, FA, FT, FTR1, FTR2, and ISNCSCI Scores in the Lesion Layer of the Observation Group

The data of ADC, FA, and FT come from the lesion layer of the observation group and the upper layer of the control group, while the data of FTR1 and FTR2 come from the lesion layer of the observation group and the middle layer of the control group. The score of ISNCSCI ranged from 225 to 341 (284.75 ± 24.89). In the observation group, ADC (*r* = −0.715, *P* < 0.001) of lesion layer was negatively correlated with ISNCSCI score, FA (*r* = 0.811, *P* < 0.001), FT (*r* = 0.664, *P* < 0.001), FTR1 (*r* = 0.571, *P* < 0.001), and FTR2 (*R* = 0.538, *P* < 0.001) were positively correlated with ISNCSCI score, see Figures 1–5.

### 3.3. Univariate Analysis of Postoperative Spinal Cord Function

Three months after the operation, JOA was used to evaluate the spinal cord function, which was excellent in 23 cases and poor in 19 cases. ISNCSCI score, ADC, FA, FT, FTR1, and FTR2 of lesion layer were all related to poor recovery of spinal cord function in patients with high cervical spinal cord tumor (*P* < 0.05), see Table 2.

### 3.4. Multivariate Analysis of Spinal Cord Function after Operation

Taking the postoperative recovery of spinal cord function of patients with high cervical spinal cord tumor as the dependent variable (see Table 3 for the assignment), and taking the items with statistically significant difference in Table 2 as the independent variable (see Table 3 for the assignment), the results were analyzed by logistic regression model. The results showed that after the ISNCSCI score was controlled, the increase in ADC and the decrease in FA, FT, FTR1, and FTR2 of the lesion layer were independent risk factors for poor postoperative body function recovery (*P* < 0.05), see Tables 3 and 4.

### 3.5. The Value of ADC, FA, FT, FTR1, and FTR2 in Lesion Layer in Predicting the Recovery of Spinal Cord Function

ROC analysis for predicting the recovery of spinal cord function after operation was drawn by taking ADC, FA, FT, FTR1, and FTR2 in focus layer of patients with poor recovery of spinal cord function as positive samples and ADC, FA, FT, and FTR2 in focus layer of patients with good recovery of spinal cord function as negative samples. The results showed that the AUC of ADC, FA, FT, FTR1, and FTR2 for predicting the recovery of spinal cord function is 0.769, 0.846, 0.813, 0.852, and 0.732, respectively. The ROC model for joint prediction of each index is constructed by applying the ROC theory model of SPSS software. The results show that the AUC of joint prediction is the largest, which is 0.941, see Figure 6 and Table 5.

## 4. Discussion

Myeloma, because the tumor oppresses the sensory and motor neurons and white matter fiber bundles of the spinal cord, often causes patients with different degrees of neurological deficits [7]. Conventional MRI can show the morphological changes of spinal cord. At present, most spinal cord tumor can be diagnosed by T1-weighted images, T2-weighted images, enhanced scans, and other sequences [8]. However, conventional MRI cannot provide information about the changes of spinal cord fine structure, which is the key to evaluate the neurological deficit of spinal cord [9]. DTI technology is currently the only noninvasive means to display the structure and course of nerve fibers. By analyzing the similarities and differences between pathological changes and normal spinal nerve anatomical structures, we can indirectly judge the relationship between lesions and gray matter and white matter of spinal cord, thus providing reference for the diagnosis, treatment, and prognosis evaluation of myeloma [10].

The spinal cord, which connects the brain with peripheral nerves, is an important organ of the central nervous system and the center of partial reflex function, in which the structure and function of white matter fiber bundle play a key role [11]. DTI technology can measure the dispersion of water molecules in tissues, show the anisotropy of dispersion movement, reflect the changes of the fine structure of spinal cord, and track the course and connection of white matter fiber bundles, so as to improve the judgment of spinal cord diseases [12]. FA and ADC are commonly used DTI parameters, in which FA is the proportion of anisotropic components of water molecules to the overall diffusion tensor, which can fully show the degree of anisotropy. ADC is a factor that can influence the movement of water molecules through calculation and reflects the intensity of water molecule dispersion movement [13]. The FT represents the number of reconstructed fiber bundles, but due to the influence of individual differences, scan resolution limitations, and so on, the FT cannot reflect the real number of white matter fibers [14]. This study introduces the calculation of FTR, that is, the ratio of FTs in different planes, which reduces the influence of software analysis and individual differences and can better reflect the damage of white matter fiber bundles [15]. This study shows that the DTI parameters FA, FT, FTR1, and FTR2 of patients with high cervical spinal cord tumor are lower than those of healthy volunteers, and the ADC is higher than that of healthy volunteers, which is basically consistent with previous studies [16]. Considering the compression of spinal cord or tumor infiltration, the structure of white matter fiber bundle is significantly affected, and the degree of anisotropy is also changed [17]. In this study, the DTI parameters of the upper layer, the lower layer, and the control group were compared, respectively, and it was found that the differences of FA, ADC, FT, and FTR mainly existed in the lower layer and the upper layer of the lesion. The analysis reason was that the compression and invasion of spinal cord tumors in the lesion layer caused the destruction of fiber bundles and involved the white matter fibers at the distal end of the lesion, resulting in fine structural changes, while the upper layer of the lesion reflected the degree of anisotropy of normal spinal cord [18]. ISNCSCI score is a commonly used score to reflect the neurological function of spinal cord, which can be used to evaluate the neurological function of patients from the aspects of motor and sensation in detail [19]. The research shows that ADC in the lesion layer of patients with high cervical spinal cord tumor is negatively correlated with ISNCCSI score, while FA, FT, FTR1, and FTR2 are positively correlated with ISNCCSI score, which indicates that DTI parameters can reflect the spinal nerve function injury of patients.

Surgical resection is the most effective treatment for high cervical spinal cord tumor. Because of the particularity of tumor location, patients are prone to hemiplegia and limb dysfunction after operation [20, 21]. Therefore, it is of great to explore the related factors that affect the spinal cord function of patients with high cervical spinal cord tumor after operation and to guide doctors to plan the operation. This study is the first time to explore the DTI parameter characteristics in the evaluation of postoperative spinal cord function. It is found that the increase in ADC and the decrease in FA, FT, FTR1, and FTR2 of the lesion layer were independent risk factors for poor postoperative body function recovery, indicate that the injury of white matter fiber bundle is more serious and the nerve function of spinal cord is worse, which is not conducive to the recovery of spinal cord function after operation. ROC analysis showed that the AUC of ADC, FA, FT, FTR1, and FTR2 in the focus layer combined to predict the recovery of spinal cord function was 0.941, which was better than that predicted separately. Therefore, the combined detection of each index can provide a more effective quantitative reference for predicting the recovery of spinal cord function in patients with high cervical spinal cord tumor after operation, so as to guide reasonable clinical treatment and improve the prognosis of patients.

To sum up, the abnormal DTI parameters of patients with high cervical myeloma can better reflect the lack of spinal cord function and can effectively predict the recovery of spinal cord function after operation, providing reference for clinical research and treatment.

## Figures and Tables

**Figure 1:** Correlation between ADC and ISNCSCI score.

**Figure 2:** Correlation between FA and ISNCSCI score.

**Figure 3:** Correlation between FT and ISNCSCI score.

**Figure 4:** Correlation between FTR1 and ISNCSCI score.

**Figure 5:** Correlation between FTR 2 and ISNCSCI score.

**Figure 6:** ROC analysis of ADC, FA, FT, FTR1, and FTR2 in the lesion layer to predict the recovery of spinal cord function.

**Table 1:** Two groups of ADC, FA, FT, and FTR ($\bar{x}\pm s$).

	ADC (×10^−9^ mm^2^/S)	FA	FT	FTR1	FTR2
Observation group (*n* = 42)					
Upper layer of lesion	1.18 ± 0.14	0.65 ± 0.05	1982.37 ± 492.39	0.76 ± 0.16^a^	0.66 ± 0.03^a^
Lesion layer	1.70 ± 0.23^a^	0.54 ± 0.13^a^	1512.43 ± 627.48^a^	1.00	1.00
Sublayer of lesion	1.30 ± 0.16^a^	0.62 ± 0.08^a^	1791.52 ± 457.76^a^	0.84 ± 0.19^a^	0.79 ± 0.21^a^
Control group (*n* = 42)					
Upper layer	1.17 ± 0.12	0.64 ± 0.04	2028.83 ± 241.46	1.00 ± 0.04	1.00 ± 0.07
Middle layer	1.15 ± 0.12	0.65 ± 0.03	2021.36 ± 268.54	1.00	1.00
Sublayer	1.16 ± 0.13	0.64 ± 0.08	1974.85 ± 309.47	1.02 ± 0.05	1.04 ± 0.06

Note: compared with the control group, ^a^*P* < 0.05.

**Table 2:** Univariate analysis of postoperative spinal cord function.

Index	Excellent (*n* = 19)	Poor (*n* = 23)	*t*/*χ*^2^	*P*
Sex				
Man	13 (68.42)	15 (65.22)	0.048	0.827
Woman	6 (31.58)	8 (34.78)		
Age (years)	42.79 ± 9.37	41.86 ± 8.64	0.334	0.740
Course of disease (months)	12.38 ± 2.85	11.86 ± 2.74	0.601	0.551
Tumor type (*n*[/%])				
Extramedullary tumor	9 (47.37)	10 (43.48)	0.064	0.801
Intramedullary tumor	10 (52.63)	13 (56.52)		
Clinical manifestation				
Limb numbness	17 (89.47)	18 (78.26)	0.308	0.579
Limb weakness	16 (84.21)	15 (65.22)	1.083	0.298
Autonomic nerve symptoms	4 (21.05)	2 (8.70)	0.485	0.486
Hoffman sign positive	5 (26.32)	2 (8.70)	1.230	0.267
Babinski sign positive	5 (26.32)	3 (13.04)	0.484	0.487
Knee hyperreflexia	4 (21.05)	2 (8.70)	0.485	0.486
ISNCSCI score (score)	265.83 ± 23.75	300.38 ± 28.63	4.198	<0.001
Layer ADC(×10^−9^ mm^2^/S)	1.85 ± 0.24	1.57 ± 0.22	3.940	<0.001
FA of lesion layer	0.45 ± 0.12	0.61 ± 0.15	3.759	<0.001
FT of lesion layer	1108.35 ± 516.37	1846.24 ± 693.57	3.838	<0.001
FTR1 of upper layer lesion	0.63 ± 0.15	0.83 ± 0.19	3.726	<0.001
FTR2 of upper layer lesion	0.67 ± 0.17	0.93 ± 0.20	4.483	<0.001

**Table 3:** Assignment.

Variable	Assignment
Dependent variable	
Recovery of spinal cord function	Excellent = 1, poor = 2
Independent variable	
ISNCSCI score	Actual value
ADC of lesion layer	Actual value
FA of lesion layer	Actual value
FT of lesion layer	Actual value
FTR1 of upper layer lesion	Actual value
FTR2 of upper layer lesion	Actual value

**Table 4:** Multivariate analysis of spinal cord function after operation.

Factor	*β*	SE	Wald *x*^2^	*P*	OR	95% CI
ADC of lesion layer	1.534	0.596	6.625	<0.001	4.635	3.058~7.026
FA of lesion layer	-0.799	0.357	5.009	0.009	0.450	0.293~0.691
FT of lesion layer	-0.826	0.332	6.190	<0.001	0.438	0.285~0.672
FTR1 of upper layer lesion	-0.721	0.324	4.952	0.025	0.486	0.319~0.741
FTR2 of upper layer lesion	-0.946	0.305	9.620	<0.001	0.388	0.254~0.593

**Table 5:** Value of ADC, FA, FT, FTR1, and FTR2 in the lesion layer in predicting the recovery of spinal cord function.

Index	AUC	95% CI	*x* ^2^	*P*	Cut-off value	Sensitivity (%)	Specificity (%)
ADC of lesion layer	0.769	0.613~0.885	3.612	<0.001	>1.71 × 10^−9^ mm^2^/S	68.42	86.96
FA of lesion layer	0.846	0.713~0.945	6.189	<0.001	≤0.63	78.65	76.52
FT of lesion layer	0.813	0.686~0.930	5.333	<0.001	≤1807.88	78.65	76.52
FTR1	0.852	0.779~0.975	9.545	<0.001	≤0.80	74.21	82.61
FTR2	0.732	0.573~0.857	2.965	<0.001	≤0.93	74.74	72.17
Union	0.941	0.822~0.990	9.809	<0.001		89.74	76.96

## Data Availability

The labeled dataset used to support the findings of this study are available from the corresponding author upon request.
